# Sentiment Analysis for Necessary Preview of 30-Day Mortality in Sepsis Patients and the Control Strategies

**DOI:** 10.1155/2021/1713363

**Published:** 2021-10-25

**Authors:** Yanqun Zou, Jian Wang, Zheng Lei, Yuanjun Zhang, Wenfeng Wang

**Affiliations:** ^1^Department of Critical Care Medicine, The First People's Hospital of Ziyang, Ziyang 641300, Sichuan, China; ^2^School of Science, Shanghai Institute of Technology, Shanghai 201418, China

## Abstract

This study was to preview the risk of 30-day mortality in sepsis patients using sentiment analysis. The clinical data of patients and nursing notes were collected from the Medical Information Mart for Intensive Care (MIMIC-III) database. The factors influencing 30-day mortality were analyzed using the Cox regression model. And, the prognostic index (PI) was estimated. The receiver operating characteristic (ROC) curve was used to determine the PI cut-off point and assess the prediction ability of the model. In total, 1844 of 3560 patients were eligible for the study, with a 30-day mortality of 37.58%. Multivariate Cox analysis showed that sentiment polarity scores, sentiment subjectivity scores, simplified acute physiology score (SAPS)-II, age, and intensive care unit (ICU) types were all associated with the risk of 30-day mortality (*P* < 0.05). In the preview of 30-day mortality, the area under the curve (AUC) of ROC was 0.78 (95%CI: 0.74–0.81,*P* < 0.001) when the cut-off point of PI was 0.467. The documented notes from nurses were described for the first time. Sentiment scores measured in nursing notes are associated with the risk of 30-day mortality in sepsis patients and may improve the preview of 30-day mortality.

## 1. Introduction

Sepsis, a complicated disorder, develops as an aberrantly regulated host response to the infection, and it is related to acute organ dysfunction and a high-risk mortality [1]. The incidence of sepsis is high, but the true incidence is unknown. A population-based study showed that the incidence of sepsis came up to 535 cases per 100,000 persons annually and was rising [2]. In two inpatient cohorts, sepsis was found to be conductive to 1 in every 2-3 deaths, and most patients were subjected to sepsis at admission [3]. Although effective measures about the prevention and treatment have been taken, and outcomes have improved, the mortality is still higher than 25%–30%, reaching up to 40%–50% when shock appears [4,5].

At present, the mortality in the intensive care unit (ICU) can be previewed by several common methods where the severity of illness scores (SOI) is often used, such as sequential organ failure assessment (SOFA), simplified acute physiology score (SAPS), and acute physiology and chronic health evaluation (APACHE) [6–8]. The SOI system is developed based on the patient's clinical data mainly obtained from the electronic health record (EHR). Nevertheless, in the common EHR, unstructured data like clinical notes are also present. There are evidences suggesting that clinicians have capabilities to reasonably predict the mortality in the ICU [9,10]. It is, thus, clear that the clinical notes written by clinicians contain valuable information on the health status of patients. As a technique of processing the natural language, sentiment analysis contributes to identifying the attitudes or impressions of clinicians towards patients through computational algorithms to extract subjective information in the written text and classify subjective properties [11–13]. Previous studies have demonstrated that there is a close association of sentiments identified in clinical notes with both hospital readmission and mortality in the ICU [14, 15].

In this study, we used a sentiment analysis method to preview the risk of 30-day mortality in sepsis patients based on Medical Information Mart for Intensive Care (MIMIC-III) database, hoping to provide more valuable information for improving the outcomes of patients in the ICU.

## 2. Methods

### 2.1. Study Design and Population

A total of 1,844 sepsis cases from the MIMIC-III database between 2001 and 2012 were enrolled in the retrospective study. The mortality from the date of ICU admission to 30 days after discharge (30-day mortality) was considered as the primary outcome of the present study. These patients were divided into the survived (*n* = 1151) and dead (*n* = 693) groups. The clinical data of patients and nursing notes were available from MIMIC-III database, a large-scale critical care database. MIMIC-III comprises information associated with the patients hospitalized in critical care units of large tertiary care hospitals, such as demographics, medications, laboratory measurements, vital signs, hospital length of stay, nursing notes, and survival data [16]. The data applied in the present study were from the MIMIC-III database (https://mimic.physionet.org/), a freely accessible database developed by the MIT Lab for Computational Physiology, comprising deidentified health data associated with −60,000 intensive care unit admissions. The data collected in the MIMIC-III was approved by the Ethics Review Board of the Beth Israel Deaconess Medical Center, and all private information has been carried out the desensitization.

Patients were screened based on the inclusion and exclusion criteria. Inclusion criteria included (1) being diagnosed as sepsis, severe sepsis, and septic shock (International Classification of Diseases 9 (ICD-9) codes: 99591, 99592, and 78552) in the MIMIC-III database and (2) having complete clinical data. Exclusion criteria incorporated (1) lack of nursing notes and (2) notes written <12 h before the death and those identified by clinicians as errors.

The diagnostic criteria of sepsis were based on Sepsis-2 [17]. Patients with sepsis were screened according to the ICD code in MIMIC-III. The ICD is presented in the form of code, which classifies diseases according to their causes, locations, pathology, and clinical manifestations, so as to realize statistical analysis, comprehensive utilization, and scientific management of diseases in hospitals. The description of nurses who had more direct contact with patients was used. Nurses can observe the early signs of deterioration in the patient's health, highlight any abnormal clinical measures, and record their judgments or concerns in their documentation. Examples are listed in Table 1. This is a retrospective study. All behaviors of medical staff were not intervened. The collection of nursing notes is a normal part of the hospital's work, so the operations of medical staff will not be affected by this study.

### 2.2. Sentiment Analysis

Sentiment is usually described as the relative polarity of a text string, with the score from −1 (very negative) to 1 (very positive) [18]. There are also other sentiment dimensions like subjectivity, emotion, and strength that can be assessed by common sentiment analysis methods [15]. In this study, Python programming language and TextBlob natural language processing library (https://textblob.readthedocs.io/en/dev/) were both used to calculate sentiment scores in the nursing notes. NLTK language processing tool was used for word segmentation; that is, nursing notes were divided into several words, and the “pattern” was used for polarity scoring to obtain several polarity scores and subjective scores. The mean of polarity scores and subjective scores was used as the final score. The sentiment polarity was returned by TextBlob as a number from −1 to 1, and the subjectivity was returned as a number from 0 to 1. The higher the scores were, the more positive and subjective the sentiment was.

### 2.3. Collection of Information

For each patient, the following information was collected, including age, gender, sentiment polarity, and subjectivity scores in nursing notes measured by sentiment analysis, SAPS-II, and ICU types. SAPS-II, a known predictor of ICU mortality, was composed of the patient's age, 12 physiology variables, 3 underlying disease variables, and admission types [19]. In the present study, it was computed based on the data accessed from MIMIC-III database and SQL scripts in the MIT Laboratory for Computational Physiology Git Repository.

### 2.4. Statistical Analysis

SPSS 22.0 software (IBM Corp., Armonk, NY, USA) and Python text analysis (version 3.7) were used to manage the data. Normally-distributed measurement data were expressed as the mean ± standard deviation ($\bar{x}\pm s$), which were compared using *t*-test; those with abnormal distribution were manifested as the median and interquartile (M (Q1, Q3)), which were compared through the Mann–Whitney U rank-sum test. *χ*^2^test was employed to compare the enumeration data manifesting as *n* (%). The influencing factors of 30-day mortality in sepsis patients were determined using the Cox regression model, and hazard ratio (HR) with 95% confidence interval (CI) was used to estimate these associations. Univariate Cox regression analysis was performed on baseline variables, and variables with statistical significance were included in the multivariate Cox regression model. The prognostic index (PI) was estimated with the formula (PI = *β*_0_ + *X*_1_*β*_1_ + *X*_2_*β*_2_ + … + *X*_*k*_*β*_*k*_). The larger the PI value, the worse the prognosis. A receiver operating characteristic (ROC) curve was drawn to determine the PI cut-off point and evaluate the preview ability of the model. SAPS-II consists of 17 factors and is not calculated using linear functions. The effect of collinearity between age and APS-II is limited, and its variance inflation factor is 1.118; thus, the effect of collinearity can be ignored. The *P* value less than 0.05 showed significant difference.

### 2.5. The Preview Model

C-statistic reflected the degree of consistency between the predictive result and actual event occurrence. In the Cox proportional hazard regression model, event occurrence could be described by whether it occurred or not and occurrence time. Therefore, for the Cox model, it was necessary to compare the actual occurrence time of the event with the event occurrence time previewed by the model to evaluate model discrimination.

For a cohort with an observation period of *t*, the actual survival time of the participants was recorded as *t*_1_, *t*_2_,… (if no event occurred until the end of the observation period, then *t*_._=*t*), and the survival time estimated by the model was recorded as *t*′, *t*_2_′,…

Then, for two different participants (*i*, *j*), the following was met:

(1) $$\begin{array}{c} t_{i}\langle t_{j}\text{ and }t^{\prime }\langle t_{j}^{\prime },\text{ or }t_{i}\rangle t_{j}\text{ and }t_{i}^{\prime }\rangle . \end{array}$$

In other words, if the inequality had the same direction, the model preview result was considered to be “consistent.”

If the inequality was in the opposite direction,

(2) $$\begin{array}{c} t_{i}\langle t_{j}\text{ and }t_{i}^{\prime }\rangle t_{j}^{\prime },\text{ or }t_{i}>t_{j}\text{ and }t_{i}^{\prime }<t_{j}^{\prime }, \end{array}$$

it was considered “inconsistent.”

If the expected survival time of the two was the same, namely,

(3) $$\begin{array}{c} t_{i}\neq t_{j},\\ t_{i}^{\prime }=t_{j}^{\prime }, \end{array}$$

it was considered “uncertain.”

In survival analysis, the survival time of an individual was difficult to preview, but there was a one-to-one corresponding relation between survival time and survival function, and the survival function could be directly calculated by the Breslow method. The survival functions of the participant at time *T* were recorded as *S*_1_, *S*_2_,… If the expected survival time of *i*(*t*_*i*_′) was longer than the expected survival time of *j*(*t*_*j*_′), then the probability of *t*_*i*_′ > *T* (*S*_*i*_) should be greater than the probability of *t*_*j*_′ > *T* (*S*_*j*_), and vice versa. At this time, formulas (1)–(3) could be rewritten as

(4) $$\begin{array}{c} \text{consistent}:\;t_{i}<t_{j}\text{ and }S_{i}\neq S_{j},\text{or }t_{i}>t_{j}\text{ and }S_{i}>S_{j},\\ \text{inconsistent}:\;t_{i}<t_{j}\text{ and }S_{i}>S_{j},\text{or }t_{i}>t_{j}\text{ and }S_{i}<S_{j},\\ \text{uncertain}:\;t_{i}\neq t_{j},\text{and }S_{i}=S_{j}. \end{array}$$

It could be seen that not every pair of participants could give an evaluation of whether it was consistent or not. When the survival time of two participants was the same, if there was no event at the end of the observation period (*t*_*i*_=*t*_*j*_=*T*), the above definition could not be used for evaluation. At this time, the pair of participants would not be taken into consideration when calculating model discrimination. In addition, for participants who were lost to follow-up or withdraw during the observation period, their survival time was not comparable to that of other participants (the life expectancy of participants censored at time *t*; was not necessarily less than that of participants who died at time *t*_*j*_ (>*t*_*j*_), so it should not be taken into consideration in the analysis.

Assuming that no participants left the cohort halfway, except for events of concern to the research, C-statistic was the consistency rate of the result predicted by the Cox proportional hazard regression model among all participants (with varying survival time) taken into consideration:

(5) $$\begin{array}{c} C=P\left(t_{i}\langle t_{j}\text{ and }S_{i}\langle S_{j},\text{ or }t_{i}\rangle t_{j}\text{ and }S_{i}\rangle S_{j}|t_{i}\neq t_{j}\right)+\frac{1}{2}P\left(S_{i}=S_{j}\right)|t_{i}\neq t_{j}. \end{array}$$

If

(6) $$\begin{array}{c} \pi_{c}=P\left(t_{i}<t_{j}\text{ and }S_{i}<S_{j}\right),\text{ or }t_{i}>t_{j}\text{ and }S_{i}>S_{j}\\ =P\left(t_{i}<t_{j}\text{ and }S_{i}<S_{j}\right)+P\left(t_{i}>t_{j}\text{ and }S_{i}>S_{j}\right),\\ \pi_{d}=P\left(t_{i}<t_{j}\text{ and }S_{i}>S_{j}\right),\text{ or }t_{i}>t_{j}\text{ and }S_{i}<S_{j}\\ =P\left(t_{i}<t_{j}\text{ and }S_{i}>S_{j}\right)+P\left(t_{i}>t_{j}\text{ and }S_{i}<S_{j}\right),\\ \pi_{u}=P\left(t_{i}\neq t_{j}\text{ and }S_{i}=S_{j}\right)\\ =P\left(t_{i}<t_{j}\text{ and }S_{i}=S_{j}\right)+P\left(t_{i}>t_{j}\text{ and }S_{i}=S_{j}\right), \end{array}$$

then *P*(*t*_*i*_ ≠ *t*_*j*_)=*π*_*c*_+*π*_*d*_+*π*_*u*_, and formula (5) could be written as follows:

(7) $$\begin{array}{c} C=\frac{\left(\pi_{c}+\left(1/2\right)\pi_{u}\right)}{\left(\pi_{c}+\pi_{d}+\pi_{u}\right)}. \end{array}$$

The unbiased estimates of *π*_*c*_, *π*_*d*_,  and   *π*_*u*_ were

(8) $$\begin{array}{c} P_{c}=\frac{1}{n\left(n-1\right)t_{i}\neq t_{j}}\sum C_{ij},\\ P_{d}=\frac{1}{n\left(n-1\right)t_{i}\neq t_{j}}\sum D_{ij},\\ P_{u}=\frac{1}{n\left(n-1\right)t_{i}\neq t_{j}}\sum U_{ij}, \end{array}$$

where *n* was the number of participants in the cohort, *n*(*n* − 1) represented the pair number of all possible participants in the case that *i* was not equal to *j* and *c*_*ij*_ took 1 when it met the definition of (4) “consistent” and took 0 in other cases. ∑*c*_*ij*_was a consistent pair number; likewise, ∑*d*_*ij*_ was an inconsistent pair number, and ∑*u*_*ij*_ was an uncertain pair number. If the pair number of all participants with unequal survival time was recorded as

(9) $$\begin{array}{c} N=\sum c_{ij}+\sum d_{ij}+\sum u_{ij}. \end{array}$$

Then, *C* could also be expressed as

(10) $$\begin{array}{c} C=\frac{\left(\sum C_{ij}+\left(1/2\right)\sum u_{ij}\right)}{N}. \end{array}$$

The 95%CI of *C* could pass the consistency rate *P*_*C*_, the inconsistency rate *P*_*d*_, and the uncertainty rate *P*_*u*_, and the following estimated the number *N* of people in the cohort:

(11) $$\begin{array}{c} \frac{w+2C}{2\left(1+W\right)}\pm \frac{\sqrt{w^{2}+4wC\left(1-C\right)}}{2\left(1+w\right)},\;\text{where }w=\frac{2z_{\alpha /2}^{2}}{n\left(p_{c}+p_{d}+p_{u}\right)}. \end{array}$$

## 3. Results

### 3.1. Baseline Information of Included Patients

In the MIMIC-III database, there were a total of 3,560 patients admitted in the ICU. In 1,128 patients without sepsis, 356 cases lacking sentiment polarity and subjectivity scores, 172 with missing SAPS-II, and 60 with missing survival data were excluded, and 1,844 cases were finally involved in the present study (Figure 1). Among these patients, 693 cases (37.58%) were dead within 30days from hospital admission to discharge. The median survival time of all included sepsis patients was 7.03 (2.53, 18.28) days. The baseline information of survived and dead patients is presented in Table 2.

Compared with the dead patients, the survived patients had higher sentiment polarity scores (*P* < 0.001) and lower SAPS-II scores (*P* < 0.001). There were significant differences between the survived and dead patients in age (*P* < 0.001) and ICU types (*P* < 0.001), but not sentiment subjectivity score, SOFA score, and gender (Table 2). The proportion distributions of the sentiment polarity score, sentiment subjectivity score, SAPS-II score, SOFA score, age, gender, and ICU types are shown in Figure 2.

The possible effects of the missing data of lacking sentiment polarity and subjectivity scores have been analyzed in Table 3. The results showed no differences in SAPS-II (*t* = 1.93, *P*=0.054), age (*χ*^*2*^ = 0.350, *P*=0.986), gender (*χ*^*2*^ = 0.015, *P*=0.901), and ICU types (*χ*^*2*^ = 2.459, *P*=0.652) between the missing and nonmissing groups. All variables were collected on the day of transferring into the ICU.

### 3.2. Univariate and Multivariate Cox Regression Analysis of 30-Day Mortality

As shown in Table 4, univariate Cox analysis indicated that the factors influencing 30-day mortality of sepsis patients included sentiment polarity scores (HR: 0.49, 95%CI: 0.44–0.54, and *P* < 0.001), sentiment subjectivity scores (HR: 0.80, 95%CI: 0.69–0.93, and *P* < 0.004), SAPS-II (HR: 1.03, 95%CI: 1.03–1.03, and*P* < 0.001), age (40–59 years, HR: 0.72, 95%CI: 0.63–0.82, and *P* < 0.001; 60–69 years, HR: 1.18, 95%CI: 1.03–1.35, and *P*=0.016; 70–79 years, HR: 1.54, 95%CI: 1.79–2.11, and *P*=0.009; ≥80 years, HR: 1.66, 95%CI: 1.48–1.86, and *P* < 0.001), and ICU types (surgical intensive care unit (SICU), HR: 0.85, 95%CI: 0.75–0.97, and *P*=0.019) (see Figure 3).

Multivariate Cox analysis showed that sentiment polarity scores (HR: 0.58, 95%CI: 0.51–0.67, and *P* < 0.001) and sentiment subjectivity scores (HR: 0.82, 95%CI: 0.71–0.94, *P* < 0.006) were both associated with a reduced risk of 30-day mortality. The risk of 30-day mortality would be increased 0.03 times when 1 point of SAPS-II score was added each time (HR: 1.03, 95%CI: 1.02–1.03, and *P* < 0.001). Compared with those aged <40years, the risk of 30-day mortality significantly increased in patients aged 40–59 (HR: 1.59, 95%CI: 1.15–2.19, and *P*=0.005), 60–69 (HR: 1.96, 95%CI: 1.41–2.72, and *P* < 0.001), 70–79 (HR: 1.55, 95%CI: 1.10–2.20, and *P*=0.013), and ≥80 years (HR: 2.1, 95%CI: 1.52–2.90, *P* < 0.001). In addition, the patients in the trauma/surgical intensive care unit (TSICU) were least likely to experience 30-day mortality compared with those in the coronary care unit (CCU) (HR: 0.52, 95%CI:0.39–0.68, and *P* < 0.001) (Table 4).

### 3.3. Preview of 30-Day Mortality in Sepsis Cases

Based on the Cox model, PI was calculated, namely, PI = 2.58–0.54 ∗ sentiment polarity − 0.2 ∗ sentiment subjectivity + 0.02 ∗  SAPS-II + 0.46 ∗ age (40–59 years) + 0.67 ∗ age (60–69 years) + 0.44 ∗ age (70–79 years) + 0.74 ∗ age (≥80 years) + 0.09 ∗ gender − 0.43 ∗ ICU type (CSRU) − 0.38 ∗ ICU type (MICU) − 0.58 ∗ ICU type (SICU) − 0.66 ∗ ICU type (TSICU). Through the ROC curve, it can be observed that the cut-off point of PI was 0.467 (Figure 4). In the preview of 30-day mortality, the diagnostic sensitivity, specificity, and the area under the curve (AUC) were 71.95%, 70.27%, and 0.78 (95%CI: 0.74–0.81, and*P* < 0.001), respectively. PI > 0.467 represented poor prognosis. The C-statistic was 0.887 (95%CI: 0.749–0.999).

## 4. Discussion

In total, 1,844 cases of sepsis were enrolled in this study, with the overall 30-day mortality of 37.58%. Multivariate Cox analysis showed that sentiment polarity scores and sentiment subjectivity scores were both statistically significant determines, even in the presence of known determines for 30-day mortality in sepsis patients. Through the ROC curve, it can be observed that the AUC of the model was 0.78 when the cut-off point of PI was 0.467, highlighting a better diagnostic accuracy in the preview of 30-day mortality. All these findings suggested that the sentiment scores measured in nursing notes were conductive to previewing the risk of 30-day mortality in sepsis patients; the nursing notes rich in information could serve as an indicator for clinical outcomes.

It is well-known that the brief fragments in the text can reflect the author's feelings on a given topic, and language processing tools are conductive to characterizing these feelings including the sentiment in text documents [20]. Sentiment, a metric usually used to explore the negative or positive opinion within messages, is weighed using a number from −1 (very negative) to 1 (very positive) [13,18]. Sentiment analysis allows the words and symbols used within a message to be checked for the intensity of negative and positive emotions and opinions [13]. In the Twitter-based healthcare research field, sentiment analysis has been the mainstream. Recently, sentiment analysis has begun to be used in the medical settings, such as encounter notes of patients with critical illness [21], and virtual visits for Parkinson's disease [22]. The studies have demonstrated that sentiment analysis can help us understand the attitudes of clinicians towards patients by categorizing the subjective expressions written in the clinical notes, thereby playing a certain role in predicting the outcomes of patients [23–25]. In this study, sentiment polarity scores and sentiment subjectivity scores were both identified as the significant determines for 30-day mortality in sepsis patients, indicating that the sentiment scores were associated with the risk of 30-day mortality. This was supported by the results concluded by McCoy et al. that higher positive sentiment at discharge was related to a notably reduced risk of hospital readmission [14]. In addition, our results also exhibited that the sentiment scores can improve the preview of 30-day mortality in sepsis patients as presented by the AUC of ROC. Hence, in the preview models of clinical outcomes, unstructured information in nursing notes should also be comprised except for traditionally used structured data [26,27].

This was the first population-based study to preview the risk of 30-day mortality in sepsis patients using sentiment analysis. The sentiment scores in nursing notes were computed using Python programming language and TextBlob natural language processing library, which was easy to operate. Moreover, our results might be more credible because the nursing notes written <12 h before the patient's death were not included. Nevertheless, some limitations in this study remained to be concerned. First, according to the mean sentiment scores, the variation in sentiment can only be characterized at the patient level instead of the clinician level. With plenty of information on clinicians, sentiment measurement would be beneficial to identification of the clinician-level factors probably affecting the outcomes. Second, the data of MIMIC-III database were obtained from a large-scaled hospital, but the nursing notes in our study only represented a part of nurses. The clinicians with different work experiences and environments may take the nursing notes with polytropic features. Third, a single-center MIMIC-III database with distinct clinical culture may affect the way of taking notes for nurses, thus leading to a limitation in generalizability of the relationship between mortality and sentiment measured in nursing notes. Text data in the health record by nurses depend on the time restraint. That is, when nurses are too busy to write for dying patients, their text information may be reduced. Therefore, more accurate sentiment measurement, biomarkers related to sepsis, and multi-center data may improve the effectiveness of models that previewed the 30-day mortality risk in sepsis patients. In addition, external validation is a necessary measure for the application of the preview model in clinical practice.

## 5. Concluding Remarks

The documented notes from nurses were described for the first time. Our results suggest that the sentiment scores measured in nursing notes are associated with the risk of 30-day mortality in sepsis patients, which may contribute to improving the preview of 30-day mortality.

## Figures and Tables

**Figure 1:** Flow chart of the patient screening.

**Figure 2:** Proportion distributions of variables between survivals and deaths in sepsis patients. (a) Sentiment polarity score; (b) sentiment subjectivity score; (c) SAPS-II score; (d) SOFA score; (e) age; (f) gender; (g) ICU types.

**Figure 3:** Associations between variables and 30-day mortality in sepsis patients.

**Figure 4:** The ROC with AUC and 95%CI for predicting 30-day mortality.

**Table 1:** Examples of nursing notes.

Examples	Description
1	Presumptive diagnosis is Lemierre given the h/o severe sore throat and neck pain followed by hypoxia as well as the CT chest c/w septic emboli in setting of growing anaerobic GNRs at the OSH. However, the CT of the neck was negative for thrombophlebitis although this is only positive in 30%–40% of cases. Other potential sources include an abdominal source given her original presentation including abdominal pain and concern for an acute abdomen. Potential alternatives include bacterial pneumonia/CAP, and atypical pneumonia, although these are less likely. TTE ruled out endocarditis as a source of septic emboli.
2	Yesterday her HCP decided to withdraw care by turning down the tidal volume, the FIO_2_ to room air, and the PEEP to 0. This was done today. She remained on 500 mcg/hr of fentanyl and 20 mg/hr of versed as well as 20 mg methadone q8hr. Her eyes were open but did not follow commands, and her limbs were flaccid.

*Note.* CT: computerized tomography; FIO_2_: fraction of inspiration O_2_; PEEP: positive end expiratory pressure.

**Table 2:** Baseline information of included patients, *n*(%) or ($\bar{x}\pm s$).

Characteristics	Survived (*n* = 1 151)	Dead (*n* = 693)
*Sentiment polarity score* ^*∗*^	0.05 ± 0.04	0.03 ± 0.04
*Sentiment subjectivity score* ^*∗*^	0.58 ± 0.04	0.38 ± 0.04
*SAPS-II* ^*∗*^	42.94 ± 15.58	56.08 ± 15.43
*SOFA score*	8.01 (6.02, 11.03)	8.08 (6.00, 11.01)

*Age* ^*∗*^ *, years*		
<40	90 (7.82)	25 (3.61)
40–59	313 (27.19)	158 (22.8)
60–69	201 (17.46)	145 (20.92)
70–79	294 (25.55)	139 (20.05)
≥80	253 (21.98)	226 (32.61)

*Gender*		
Female	524 (45.53)	301 (43.43)
Male	627 (54.47)	392 (56.57)

*ICU types* ^*∗*^		
CCU	45 (3.91)	54 (7.79)
CSRU	32 (2.78)	29 (4.18)
MICU	653 (56.73)	432 (62.34)
SICU	265 (23.02)	113 (16.31)
TSICU	156 (13.55)	65 (9.38)

*Note.* ^*∗*^ *P* < 0.05. SAPS-II: simplified acute physiology score II; SOFA: sequential organ failure assessment; ICU: intensive care unit; CCU: coronary care unit; CSRU: cardiac surgery recovery unit; MICU: medical intensive care unit; SICU: surgical intensive care unit; TSICU: trauma/surgical intensive care unit.

**Table 3:** Difference analysis between the missing and nonmissing data, *n* (%) or ($\bar{x}\pm s$).

Variables	Missing (*n* = 356)	Nonmissing (*n* = 1844)	Statistics	*P*
*SAPS-II*	46.63 ± 17.21	45.45 ± 16.15	*t* = 1.93	0.054
*SOFA*	8.00 (6.01, 11.00)	8.04 (5.95, 11.08)	*Z* = 1.637	0.102

*Age, years*			*χ* ^*2*^ = 0.350	0.986
<40	22 (6.15)	115 (6.24)		
40–59	87 (24.56)	471 (25.54)		
60–69	70 (19.53)	346 (18.76)		
70–79	86 (24.06)	433 (23.48)		
≥80	91 (25.70)	479 (25.98)		

*Gender*			*χ* ^*2*^ = 0.015	0.901
Female	158 (44.44)	825 (44.74)		
Male	198 (55.56)	1019 (55.26)		

*ICU type*			*χ* ^*2*^ = 2.459	0.652
CCU	14 (4.01)	99 (5.37)		
CSRU	15 (4.18)	61 (3.31)		
MICU	213 (59.84)	1085 (58.84)		
SICU	68 (19.00)	378 (20.50)		
TSICU	46 (12.97)	221 (11.98)		

*Note*. SAPS-II: simplified acute physiology score II; ICU: intensive care unit; CCU: coronary care unit; CSRU: cardiac surgery recovery unit; MICU: medical intensive care unit; SICU: surgical intensive care unit; TSICU: trauma/surgical intensive care unit.

**Table 4:** Univariate and multivariate Cox regression analysis of 30-day mortality.

Variables	Univariate analysis		Multivariate analysis		
	HR (95%CI)	*P*	HR (95%CI)	*P*	*β*
*Sentiment polarity score*	0.49 (0.44–0.54)	<0.001	0.58 (0.51–0.67)	<0.001	−0.54
*Sentiment subjectivity score*	0.80 (0.69–0.93)	0.004	0.82 (0.71–0.94)	0.006	−0.20
*SAPS-II*	1.03 (1.03–1.03)	<0.001	1.03 (1.02–1.03)	<0.001	0.02
*SOFA*	1.01 (0.99–1.03)	0.278	1.01 (0.98–1.03)	0.283	0.01

*Age (<40), years*					
40–59	0.72 (0.63–0.82)	<0.001	1.59 (1.15–2.19)	0.005	0.46
60–69	1.18 (1.03–1.35)	0.016	1.96 (1.41–2.72)	<0.001	0.67
70–79	1.54 (1.79–2.11)	0.009	1.55 (1.10–2.20)	0.013	0.44
≥80	1.66 (1.48–1.86)	<0.001	2.1 (1.52–2.90)	<0.001	0.74

*Gender (female)*					
Male	1.08 (0.97–1.20)	0.142	1.09 (0.98–1.22)	0.102	0.09

*ICU types (CCU)*					
CSRU	1.02 (0.76–1.37)	0.902	0.65 (0.45–0.94)	0.021	−0.43
MICU	1.10 (0.99–1.22)	0.091	0.69 (0.54–0.87)	0.002	−0.38
SICU	0.85 (0.75–0.97)	0.019	0.56 (0.43–0.73)	<0.001	−0.58
TSICU	0.89 (0.76–1.04)	0.153	0.52 (0.39–0.68)	<0.001	−0.66

*Note*. HR: hazard ratio; 95%CI: 95% confidence interval; SAPS-II: simplified acute physiology score II; sequential organ failure assessment; ICU: intensive care unit; CCU: coronary care unit; CSRU: cardiac surgery recovery unit; MICU: medical intensive care unit; SICU: surgical intensive care unit; TSICU: trauma/surgical intensive care unit.

## Data Availability

The data applied in the present study were from the MIMIC-III database (https://mimic.physionet.org/), a freely accessible database developed by the MIT Lab for Computational Physiology, comprising deidentified health data associated with 60,000 intensive care unit admissions.
